The article "Gyroscope Sensor Based In Vivo Finger Axes of Rotation Identification Using Screw Displacement" was published in 2021. Journal: Appl Bionics Biomech.

# Gyroscope Sensor Based *In Vivo* Finger Axes of Rotation Identification Using Screw Displacement

**DOI:** 10.1155/2021/8871593

**Published:** 2021-02-10

**Authors:** Yiming Zhu, Guowu Wei, Lei Ren, Zirong Luo, Jianzhong Shang

**Affiliations:** ^1^School of Mechanical, Aerospace and Civil Engineering, The University of Manchester, Manchester, M13 9PL, UK; ^2^School of Mechatronics Engineering and Automation, National University of Defence Technology, 410073, China; ^3^School of Science, Engineering and Environment, University of Salford, Salford, M5 4WT, UK

## Abstract

This paper presents a low-cost, efficient, and portable *in vivo* method for identifying axes of rotation of the proximal interphalangeal and distal interphalangeal joints in an index finger. The approach is associated with the screw displacement representation of rigid body motion. Using the matrix exponential method, a detailed derivation of general spatial displacement of a rigid body in the form of screw displacement including the Rodrigues' formulae for rotation is presented. Then, based on a gyroscope sensor, a test framework for determining axes of rotation of finger joints is established, and experiments on finding the directions of joint axes of the PIP and DIP joints are conducted. The results obtained highly agree with those presented in literature through traditional but complex methods.

## 1. Introduction

For clinical, prosthetic, rehabilitation, and ergonomic applications, an accurate model of the kinematics of the joints in the fingers is essential for better understanding their normal function and pathology. The axes of rotation of the finger joints are crucial in the kinematic modelling and have great impact on muscle activation. Hence, knowledge of their location and orientation is important for constructing prosthetic joints and in the planning of reconstructive surgeries like tendon transfers [1]. So far, several different methods have been proposed for identifying the axes of rotation in human hand joints. These include the mechanical approach by using an “axis finder” to find axes of rotation in the thumb and index finger metacarpophalangeal (MCP) joints and the thumb carpometacarpal (CMC) and interphalangeal (IP) joints [2, 3]; the MR image-based method for modelling the proximal interphalangeal (PIP) and distal interphalangeal (DIP) joint kinematics [4]; the CT image-based method for identifying the trapeziometacarpal joint during thumb extension/flexion and abduction/adduction [5]; the LED and CT-based cadaveric investigation for PIP joint of an index finger [6]; and the surface marker-based method for thumb carpometacarpal joint kinematics [7], for determination of the centre of rotations (CORs) of the DIP, PIP, and MCP joints in the four fingers [8], and for identification of centres and axes of rotation of wrist and fingers in hand kinematic modelling [9]. Except for the “axis finder,” the approaches presented previously are costly and complex. However, the “axis finder” is based on the assumption that the finger joint axis is fixed and can only approximately find the rotation axis of a joint at one specified position per measurement. Hence, the “axis finder” cannot provide continuous measurement for the whole range of motion of a finger joint and thus the accurate vector of the average rotation axis.

In this paper, we propose an economic, intuitive, and portable measuring method based on gyroscope sensors. We show that combine with the screw displacement representation of rigid body motion, the proposed method is efficient for finding the axes of rotation of the PIP and DIP joints, and for presenting kinematics of the middle and distal phalanges in an index finger. The finger joints are formed by bones which are commonly treated as rigid bodies, and, hence, the classical rigid body motion representation methods can be used to describe the motion of bones and the associated joints. Considering the motion of bones as general spatial displacement, we introduce screw displacement representation [10] to present the motion of joints and bones in fingers. Screw displacement is widely used in the fields of kinematics, robotics, and computer vision but is not very popular in the field of biomechanics. To formulate the screw displacement, there are mainly two approaches, one based on geometric and vector interpretation and the other with exponential derivation [11–14]. It is a very useful and effective tool for identifying axes of rotation of joints and presenting kinematics of fingers [15]. Hence, the detailed derivation of screw displacement of rigid body motion is presented in detail in this paper.

This paper firstly presents the matrix-exponential-based representation of screw displacement of rigid body motion laying background for the derivation and identification of axes of rotation of finger joints. Then, a low-cost gyroscope-sensor-based solution is proposed to identify the direction vectors of the PIP and DIP joint axes in an index finger, providing an *in vivo* method for determining axes of rotation of finger joints. Discussions of the results and limits are addressed, and a conclusion is drawn.

## 2. Screw Displacement Representation of Rigid Body Motion

In the human hand, bones are responsible for rigidity and joints between the bones provide freedom of movement. Hence, assuming no deformation, motions among the bones in the hand can be treated as rigid body motion. According to Chasles' theorem [10], the general motion between two rigid bodies is screw motion as presented in exponential derivation of this section [11].

### 2.1. Exponential Derivation for Rotation

Rotation and translation combined leads to the general spatial motion of a rigid body in the three-dimensional space. There are cases that motion between two bodies is a pure rotation which can be mathematically presented with a rotation matrix **R** that belongs to the special orthogonal group as **R** ∈ SO(3). Referring to Figure 1, we find that the rotation matrix can be expressed as a function of rotation angle *θ* and a vector **ω** that presents the direction of the axis of rotation.

Figure 1 shows the rotation of rigid body 1 with respect to body 0 about an axis passing through point *O* in the direction **ω** which is coincident with the *z*-axis of a reference frame *O* − *xyz*. If the rigid body rotates at a constant unit angular velocity about the axis **ω**, the velocity of a point *P* on the body, denoted as $\dot{p}$, can be expressed as

(1) $$\begin{array}{c} \dot{p}\left(t\right)=\omega \times p\left(t\right)=\left[\omega \right]p\left(t\right), \end{array}$$

where [**ω**] is the skew-symmetric matrix representation for the cross product of vector **ω**, which complies with [**ω**]^*T*^ = −[**ω**]. Equation (1) is a time-invariant differential equation which can be integrated resulting in

(2) $$\begin{array}{c} p\left(t\right)=e^{\left[\omega \right]t}p\left(0\right), \end{array}$$

with **p**(0) and **p**(*t*) being the initial (at time *t* = 0) and current (at time *t*) positions of point *P*, respectively (see Figure 1), and the matrix exponential *e*^[**ω**]*t*^ can be expressed in Taylor's series form as

(3) $$\begin{array}{c} e^{\left[\omega \right]t}=I+\left[\omega \right]t+\frac{{\left[\omega \right]}^{2}t^{2}}{2!}+\frac{{\left[\omega \right]}^{3}t^{3}}{3!}+\cdots , \end{array}$$

where **I** is a 3 × 3 identity matrix. Assuming that the rotation about axis **ω** is a rotation with unit angular velocity for *θ* units of time, *e*^[**ω**]*t*^ becomes *e*^[**ω**]*θ*^, and Eq. (3) thus becomes

(4) $$\begin{array}{c} e^{\left[\omega \right]\theta }=\exp\left(\left[\omega \right]\theta \right)=I+\left[\omega \right]\theta +\frac{{\left[\omega \right]}^{2}\theta^{2}}{2!}+\frac{{\left[\omega \right]}^{3}\theta^{3}}{3!}+\cdots . \end{array}$$

Considering the relations that [**ω**]^2^ = **ωω**^*T*^ − ‖**ω**‖**I**, [**ω**]^3^ = −‖**ω**‖^2^[**ω**], and ‖**ω**‖ = 1, Eq. (4) can be further expended as

(5) $$\begin{array}{c} e^{\left[\omega \right]\theta }=I+\theta \left[\omega \right]+\frac{\theta^{2}}{2!}{\left[\omega \right]}^{2}-\frac{\theta^{3}}{3!}\left[\omega \right]-\frac{\theta^{4}}{4!}{\left[\omega \right]}^{2}+\frac{\theta^{5}}{5!}\left[\omega \right]+\frac{\theta^{6}}{6!}{\left[\omega \right]}^{2}-\frac{\theta^{7}}{7!}\left[\omega \right]-\frac{\theta^{8}}{8!}{\left[\omega \right]}^{2}+\cdots =I+\left(\theta -\frac{\theta^{3}}{3!}+\frac{\theta^{5}}{5!}-\frac{\theta^{7}}{7!}+\cdots \right)\left[\omega \right]+\left(\frac{\theta^{2}}{2!}-\frac{\theta^{4}}{4!}+\frac{\theta^{6}}{6!}-\frac{\theta^{8}}{8!}+\cdots \right){\left[\omega \right]}^{2}. \end{array}$$

Using the relations that *θ* − *θ*^3^/3!+*θ*^5^/5!−*θ*^7^/7!+⋯ = sin*θ* and *θ*^2^/2!−*θ*^4^/4!+*θ*^6^/6!−*θ*^8^/8!+⋯ = 1 − cos*θ*, Eq. (5) can be simplified as

(6) $$\begin{array}{c} e^{\left[\omega \right]\theta }=I+\sin\theta \left[\omega \right]+\left(1-\cos\theta \right){\left[\omega \right]}^{2}=\cos\theta I+\sin\theta \left[\omega \right]+\left(1-\cos\theta \right){\omega \omega }^{T}. \end{array}$$

Equation (6) is known as Rodrigues' formula for a rotation of a rigid body about an arbitrary axis passing through the origin of a reference coordinate system. It is a rotation matrix which can also be obtained through the geometric method [15]. Hence, expending Eq. (6) leads to a rotation matrix

(7) $$\begin{array}{c} R\left(\left[\omega \right],\theta \right)=e^{\left[\omega \right]\theta }=I+\sin\theta \left[\omega \right]+\left(1-\cos\theta \right){\left[\omega \right]}^{2}=\left[\begin{array}{ccc} r_{11} & r_{12} & r_{13}\\ r_{21} & r_{22} & r_{23}\\ r_{31} & r_{32} & r_{33} \end{array}\right], \end{array}$$

where with the joint axis vector being **ω** = [*ω*_*x*_, *ω*_*y*_, *ω*_*z*_]^*T*^, the elements *r*_*ij*_ in Eq. (7) are as follows: *r*_11_ = cos*θ* + *ω*_*x*_^2^(1 − cos*θ*), *r*_12_ = *ω*_*x*_*ω*_*y*_(1 − cos*θ*) − *ω*_*z*_sin*θ*, *r*_13_ = *ω*_*x*_*ω*_*z*_(1 − cos*θ*) + *ω*_*y*_sin*θ*, *r*_21_ = *ω*_*y*_*ω*_*x*_(1 − cos*θ*) + *ω*_*z*_sin*θ*, *r*_22_ = cos*θ* + *ω*_*y*_^2^(1 − cos*θ*), *r*_23_ = *ω*_*y*_*ω*_*z*_(1 − cos*θ*) − *ω*_*x*_sin*θ*, *r*_31_ = *ω*_*z*_*ω*_*x*_(1 − cos*θ*) − *ω*_*y*_sin*θ*, *r*_32_ = *ω*_*z*_*ω*_*y*_(1 − cos*θ*) + *ω*_*x*_sin*θ*, and *r*_33_ = cos*θ* + *ω*_*z*_^2^(1 − cos*θ*).

Hence, substituting Eq. (7) into Eq. (2) implies that *e*^[**ω**]*t*^**p**(0) has the effect of rotating point *P* about a fixed axis **ω** by an angle *θ* to a new position **p**(t).

Equation (7) is also known as the screw-axis representation of the rotation of a rigid body. Such a representation involves four parameters: three describing the direction of the screw (joint axis) and one associated with the angle of rotation, whereas only two of the three variables giving the direction of the screw axis are independent because they comply with the condition of a unit vector, i.e., *ω*_*x*_^2^ + *ω*_*y*_^2^ + *ω*_*z*_^2^ = 1.

Equation (7) indicates that for any rotation motion, there always exists an instantaneous axis **ω** about which the rotation is associated together with the angle *θ*. Hence, given the joint axis vector and the angle of rotation, the nine elements of the rotation matrix in Eq. (7) can be computed. On the other hand, given a rotation matrix **R**, the vector of joint axis (screw axis) **ω** and the angle of rotation *θ* can be calculated. Observing the elements in the rotation matrix in Eq. (7), the angle of rotation *θ* can be obtained by adding the diagonal elements of the rotation matrix as

(8) $$\begin{array}{c} \theta =\cos^{-1}\left(\frac{\text{tr}R-1}{2}\right)=\cos^{-1}\left(\frac{r_{11}+r_{22}+r_{33}-1}{2}\right), \end{array}$$

where tr**R** stands for the trace of matrix **R** and tr**R** = *r*_11_ + *r*_22_ + *r*_33_ = 1 + 2cos*θ*.

Further investigating the rotation matrix, direction of the screw axis can be obtained by taking the differences between each pair of the two opposing off-diagonal elements:

(9) $$\begin{array}{c} \omega =\left[\begin{array}{c} \omega_{x}\\ \omega_{y}\\ \omega_{z} \end{array}\right]=\frac{1}{2\sin\theta }\left[\begin{array}{c} r_{32}-r_{23}\\ r_{13}-r_{31}\\ r_{21}-r_{12} \end{array}\right]. \end{array}$$

If represented in the skew-symmetric form, [**ω**] can also be expressed as

(10) $$\begin{array}{c} \left[\omega \right]=\left[\begin{array}{ccc} 0 & -\omega_{z} & \omega_{y}\\ \omega_{z} & 0 & -\omega_{x}\\ -\omega_{y} & \omega_{x} & 0 \end{array}\right]=\frac{\left(R-R^{T}\right)}{2\sin\theta }. \end{array}$$

Since the angle *θ* in Eq. (8) has either positive or negative value, Eqs. (9) and (10) give two solutions of the screw axis, one being the negative of the other. However, the two solutions represent the same screw since a rotation of angle −*θ* about axis −**ω** has the same result as a rotation of *θ* about the **ω** axis.

### 2.2. Exponential Expression of Spatial Rigid-Body Motion

Section 2.1 presents the exponential derivation of rotation motion of a rigid body. The same process can be applied to derive the general spatial motion of a rigid body in the three-dimensional space. Chasles' theorem states that general motion of a rigid body in three-dimensional space is a rotation and a translation long some axis, such a motion is known as a screw displacement [16].

Figure 2 shows the motion of a point *P* on a rigid body from *P*_1_ firstly to *P*_2_^*r*^ and then to *P*_2_, and the motion contains a rotation by *θ* and a translation by *d*, respectively, around and along a axis **ω**. The combination of the two motions is a screw motion about axis **ω**, with direction of the axis given by a unit vector $\omega ={\left[\begin{array}{ccc} \omega_{x} & \omega_{y} & \omega_{z} \end{array}\right]}^{T}$. By analogizing the motion with the motion of a screw, if the angle *θ* ≠ 0, pitch of the screw can be defined as *h* = *d*/*θ* such that the net translation after a rotation by *θ* is *hθ*. The two variables *θ* and *d* are screw parameters which together with the screw axis **ω** completely define the general displacement of a rigid body in the three-dimensional space.

Referring to Figure 2, **ω** is the axis direction with ‖**ω**‖ = 1, and **r**_0_ is the vector for a point *R*_0_ on the axis. Let the rigid body rotate about axis **ω** by an angular velocity of $\dot{\theta }\omega$ together with a translational velocity of $\dot{d}\omega =h\dot{\theta }\omega$, and the velocity of point *P* at **p**(*t*) can be written as

(11) $$\begin{array}{c} \dot{p}\left(t\right)=\omega \times \left(p\left(t\right)-r_{0}\right)+h\omega . \end{array}$$

This equation can be represented in a homogeneous matrix form as

(12) $$\begin{array}{c} \left[\begin{array}{c} \dot{p}\\ 0 \end{array}\right]=\left[\begin{array}{cc} \left[\omega \right] & -\omega \times r_{0}+h\omega \\ 0 & 0 \end{array}\right]\left[\begin{array}{c} p\\ 1 \end{array}\right]=\left[\begin{array}{cc} \left[\omega \right] & v\\ 0 & 0 \end{array}\right]\left[\begin{array}{c} p\\ 1 \end{array}\right]=\left[S\right]\left[\begin{array}{c} p\\ 1 \end{array}\right], \end{array}$$

where **v** = −**ω** × **r**_0_ + *h ***ω**, and hence, there exists

(13) $$\begin{array}{c} \dot{\bar{p}}\left(t\right)=\left[S\right]\bar{p}\left(t\right). \end{array}$$

Similar to solving the rotation case in Eq. (1), Eq. (13) can be solved as

(14) $$\begin{array}{c} \bar{p}\left(t\right)=e^{\left[S\right]t}\bar{p}\left(0\right), \end{array}$$

where the matrix exponential of matrix [**S**] can be derived with Taylor's series as

(15) $$\begin{array}{c} e^{\left[S\right]t}=I+\left[S\right]t+\frac{{\left(\left[S\right]t\right)}^{2}}{2!}+\frac{{\left(\left[S\right]t\right)}^{3}}{3!}+\cdots , \end{array}$$

and if assuming that the rigid body rotates about axis **ω** at a unit velocity for *θ* units of time, Eq. (15) becomes

(16) $$\begin{array}{c} T=e^{\left[S\right]\theta }=I+\left[S\right]\theta +{\left[S\right]}^{2}\frac{\theta^{2}}{2!}+{\left[S\right]}^{3}\frac{\theta^{3}}{3!}+\cdots , \end{array}$$

with ${\left[S\right]}^{2}=\left[\begin{array}{cc} {\left[\omega \right]}^{2} & v\\ 0 & 0 \end{array}\right]$, ${\left[S\right]}^{3}=\left[\begin{array}{cc} {\left[\omega \right]}^{3} & {\left[\omega \right]}^{2}v\\ 0 & 0 \end{array}\right]$, ${\left[S\right]}^{4}=\left[\begin{array}{cc} {\left[\omega \right]}^{4} & {\left[\omega \right]}^{3}v\\ 0 & 0 \end{array}\right]$,

And, hence, considering Eqs. (5) and (6), it has

(17) $$\begin{array}{c} T=e^{\left[S\right]\theta }=\left[\begin{array}{cc} e^{\left[\omega \right]\theta } & Q\left(\theta \right)v\\ 0 & 1 \end{array}\right]=\left[\begin{array}{cc} R & q\\ 0 & 1 \end{array}\right], \end{array}$$

where the term **Q**(*θ*) is

(18) $$\begin{array}{c} Q\left(\theta \right)=I\theta +\left[\omega \right]\frac{\theta^{2}}{2!}+{\left[\omega \right]}^{2}\frac{\theta^{3}}{3!}+{\left[\omega \right]}^{3}\frac{\theta^{4}}{4!}+\cdots =I\theta +\left(\frac{\theta^{2}}{2!}-\frac{\theta^{4}}{4!}+\frac{\theta^{6}}{6!}-\cdots \right)\left[\omega \right]+\left(\frac{\theta^{3}}{3!}-\frac{\theta^{5}}{5!}+\frac{\theta^{7}}{7!}-\cdots \right){\left[\omega \right]}^{2}=I\theta +\left(1-\cos\theta \right)\left[\omega \right]+\left(\theta -\sin\theta \right){\left[\omega \right]}^{2}. \end{array}$$

Using the identities that [**ω**]^2^**ω** = 0 and [**ω**]^3^ = −[**ω**], and with **v** = −**ω** × **r**_0_ + *h ***ω**, the term **Q**(*θ*)**v** can be derived as

(19) $$\begin{array}{c} Q\left(\theta \right)v=\left[I\theta +\left(1-\cos\theta \right)\left[\omega \right]+\left(\theta -\sin\theta \right){\left[\omega \right]}^{2}\right]\left(-\omega \times r_{0}+h\omega \right)=I\theta \left(-\omega \times r_{o}+h\omega \right)+\left(1-\cos\theta \right)\left[\omega \right]\left(-\omega \times r_{0}+h\omega \right)+\left(\theta -\sin\theta \right){\left[\omega \right]}^{2}\left(-\omega \times r_{0}+h\omega \right)=-\left[\omega \right]r_{0}\theta +h\theta \omega -\left(1-\cos\theta \right){\left[\omega \right]}^{2}r_{0}+0+\left(\theta -\sin\theta \right)\left[\omega \right]r_{0}+0=h\theta \omega -\left(1-\cos\theta \right){\left[\omega \right]}^{2}r_{0}-\sin\theta \left[\omega \right]r_{0}=\left(I-e^{\left[\omega \right]\theta }\right)r_{0}-h\theta \omega =\left(I-R\right)r_{0}-d\omega =q. \end{array}$$

Expending Eq. (19) gives

(20) $$\begin{array}{c} q=\left[\begin{array}{c} q_{x}\\ q_{y}\\ q_{z} \end{array}\right]=\left[\begin{array}{c} d\omega_{x}-r_{0x}\left(r_{11}-1\right)-r_{0y}r_{12}-r_{0z}r_{13}\\ d\omega_{y}-r_{0x}r_{21}-r_{0y}\left(r_{22}-1\right)-r_{0z}r_{23}\\ d\omega_{z}-r_{0x}r_{31}-r_{0y}r_{32}-r_{0z}\left(r_{33}-1\right) \end{array}\right]. \end{array}$$

Substituting Eq. (19) into Eq. (17), the transformation matrix **T** becomes

(21) $$\begin{array}{c} T=e^{\left[\omega \right]\theta }=\left[\begin{array}{cc} R & q\\ 0 & 1 \end{array}\right]=\left[\begin{array}{cc} e^{\left[\omega \right]\theta } & \left(I-e^{\left[\omega \right]\theta }\right)r_{0}+h\theta \omega \\ 0 & 1 \end{array}\right]=\left[\begin{array}{cc} R & \left(I-R\right)r_{0}+d\omega \\ 0 & 1 \end{array}\right]. \end{array}$$

In addition, using the relation that **ω**^*T*^**v** = **ω**^*T*^(−**ω** × **r**_0_) + *h ***ω**^*T*^**ω** such that *h* = **ω**^*T*^**v** and **r**_0_ = **ω** × **v**, Eq. (21) can also be expressed as

(22) $$\begin{array}{c} T=e^{\left[\omega \right]\theta }=\left[\begin{array}{cc} e^{\left[\omega \right]\theta } & \left(I-e^{\left[\omega \right]\theta }\right)\left(\omega \times v\right)+{\omega \omega }^{T}v\theta \\ 0 & 1 \end{array}\right]=\left[\begin{array}{cc} e^{\left[\omega \right]\theta } & \left[\left(I-e^{\left[\omega \right]\theta }\right)\left[\omega \right]+{\omega \omega }^{T}\theta \right]v\\ 0 & 1 \end{array}\right]. \end{array}$$

In the case that the motion is pure translation with ‖**ω**‖ = 0 and ‖**v**‖ = 1, it has **R** = *e*^[**ω**]*θ*^ = **I** such that

(23) $$\begin{array}{c} T=e^{\left[S\right]\theta }=\left[\begin{array}{cc} I & dv\\ 0 & 1 \end{array}\right]. \end{array}$$

On the other hand, in the case that the motion is pure rotation with *h* = *d* = 0 and ‖**ω**‖ = 1, it has

(24) $$\begin{array}{c} T=e^{\left[S\right]\theta }=\left[\begin{array}{cc} e^{\left[\omega \right]\theta } & \left(I-e^{\left[\omega \right]\theta }\right)r_{0}\\ 0 & 1 \end{array}\right]=\left[\begin{array}{cc} e^{\left[\omega \right]\theta } & \left(I-e^{\left[\omega \right]\theta }\right)\left(\omega \times v\right)\\ 0 & 1 \end{array}\right]. \end{array}$$

In the above equations **r**_0_ = [*r*_0*x*_ *r*_0*y*_ *r*_0*z*_]^*T*^ is a vector for a point on the screw axis and is perpendicular to the axis (see Figure 2).

There are eight parameters required in the above derivation of a spatial displacement, three for presenting direction of the screw axis **ω**, three for locating of the screw axis, i.e., **r**_0_, one for the rotation angle *θ*, and one for the translational distance *d*. However, the three parameters relative to the direction of screw axis must comply with **ω**^*T*^**ω** = 1, and, hence, only two of them are independent. In addition, only two of the three parameters that depict location of the screw axis are independent, since there exits the relationship that **r**_0_^*T*^ **ω** = 0. In summary, only six of the eight parameters are independent.

Therefore, from the above derivation, given the six parameters for describing the screw axis and the associated variables, the transformation matrix for spatial displacement in Eqs. (21) and (22) can be obtained. On the other hand, providing a specified spatial displacement of a rigid body with a rotation matrix **R** and a position vector **q**, angle of rotation *θ* can be found using Eq. (8), direction of the screw axis can be solved with Eq. (9) or Eq. (10), and the translational displacement *d* can be calculated with

(25) $$\begin{array}{c} d=\frac{\omega^{T}q}{{\left\|\omega \right\|}^{2}}. \end{array}$$

Since these equations are linear, there exists one solution corresponding to each solution set of **ω**, *θ*, and *d*.

The screw displacement form of general spatial motion derived above lays background for the kinematic analysis of robot manipulator with transform operator approach [17], which is also known as POE (product of exponential) method [13]. The POE presentation of robotic kinematics is different from the Denavit-Hartenberg convention [18] in the setting of coordinate frames and system variables. In this paper, the screw displacement approach presented above is used in the identification and representation of joint axes of rotation of human fingers.

## 3. Gyroscope Sensor-Based *In Vivo* Finger Joint Axis Identification

The axis of rotation between two bones is loosely defined as a line that does not move with respect to either bone while the bones move around each other [1]. Identifying finger join axis is important in constructing prosthetic joints and in planning reconstructive surgery of human finger. In this section, a novel and efficient method is presented for *in vivo* finger joint axis identification.

### 3.1. Representation of Joint Axis Using Screw Displacement

A human finger contains three phalanges connected by three joints including the metacarpophalangeal (MCP) joint, proximal interphalangeal (PIP) joint, and distal interphalangeal (DIP) joint. Actuated by extrinsic and intrinsic muscles (six or seven for the fingers and eight for the thumb), the fingers can perform agile movement leading to the grasping and dexterous manipulation of human hand. In the kinematic modelling of the fingers, it is commonly assumed that the joint axes of the PIP and DIP joints are parallel to each other and perpendicular to the sagittal plane. However, these assumptions are not accurate since the joint axes in human finger have neither parallel nor perpendicular relationships. The joint axes are formed according to the shapes of the bones, leading to the so-called conjoint rotations of the joints and the three-dimensional movements of the fingers [1, 20]. As pointed out in [1], the joint axes are assumed to be fixed with respect to the associated phalanges and can be identified with various methods [2–8]. This paper proposes a low-cost and efficient method for identifying the axes of DIP and PIP joints in the fingers. The proposed method is related to the screw displacement representation derived in Section 2.

Figure 3(a) shows a finger with three coordinate frames {*O*_*p*_}, {*o*_*m*_}, and {*o*_*d*_} attached to the centres of the head of the proximal, middle, and distal phalanges, respectively. At the anatomical position, as shown in Figure 3(a), the orientations of frames {*O*_*p*_}, {*o*_*m*_}, and {*o*_*d*_} are coincident. The frames are defined in such a manner of the *x*-axis is along the radial-ulnar direction, the *y*-axis is along the proximal-distal direction, and the *z*-axis is along the dorsal-palmar direction. Taking the motion of the middle phalanx about the PIP joint with respect to the proximal phalanx as an example, referring to Figure 3(b), if the middle phalanx rotates from position 1 (at anatomical position such that frame {*o*_*m*_} aligns with frame {*O*_*p*_}) to position 2, with respect to frame {*O*_*p*_}, the change of orientation of the middle phalanx, which is reflected in orientation change of frame {*o*_*m*_}, can be expressed in a rotation matrix of direction cosine form [13] as

(26) R21=xp·xm2xp·ym2xp·zm2yp·xm2yp·ym2yp·zm2zp·xm2zp·ym2zp·zm2.

With this rotation matrix and considering the relation that _2_^1^**R** = **R**(**ω**, *θ*), using Eq. (8) and Eq. (9) or (10), the joint axis about which the middle phalanx rotating with respect to the proximal phalanx **ω** and the rotating angle *θ* (see Figure 3(b)) can be calculated as

(27) θ=cos−1trR21−12=cos−1xp·xm2+yp·ym2+zp·zm2−12

and

(28) ω=0−ωzωyωz0−ωx−ωyωx0=12sinθR21−R21T.

Therefore, once the rotation matrix in Eq. (26) is given, the rotation angle *θ* and the joint axis $\omega ={\left[\begin{array}{ccc} \omega_{x} & \omega_{y} & \omega_{z} \end{array}\right]}^{T}$ can be obtained, since rotation of the middle phalanx about joint axis **ω** relative to the proximal phalanx takes a sequence of positions and thus a sequence of rotation matrices _2_^1^**R**_*i*_, leading to sequence of rotation angle *θ*_*i*_ and joint axis vector **ω**_*i*_. Hence, the direction of joint axis of the PIP joint can be obtained by taking the average of the net values as

(29) $$\begin{array}{c} \bar{\omega }=\frac{1}{n}\overset{n}{\underset{i=1}{\sum }}\omega_{i}. \end{array}$$

From the above derivation, it can be found that the key to identify the direction of joint axis is the rotation matrix **R**. In this paper, an efficient, intuitive and *in vivo* method is presented for finding **R** and thus direction of join axis based on a gyroscope sensor.

### 3.2. Gyroscope Sensor-Based *In Vivo* Finger Joint Axis of Rotation Detection

In this section, the MPU-9250 gyroscope sensor (Banggood Technology, Cyprus) is used for *in vivo* identification of joint axes of the PIP and DIP joints. As shown in Figure 4, for testing the PIP joint rotation axis of an index finger, two MPU-9250 sensors were attached to the proximal and middle phalanges, respectively, which are both connected to the Arduino board (Mega2560, ARDUINO), providing the orientation information for both the proximal and middle phalanges. During the test, the proximal phalanx is fixed, and we move the middle phalanx in an even sequence. Data containing orientation information of both the two surface gyroscopes is collected at each motion step of the middle phalanx. Then, through the open source programme from the SparkFun Electronics and the filter algorithm developed by Sebastian Madgwick of the University of Bristol, the raw data gathered from the MPU-9250 gyroscopes can be transformed and output as quaternion groups, which can be further transformed into the direction cosine matrix **R** in computer programme such as MATLAB®. It should be pointed out that the hand does not have to be in a prone position (see Figure 4) for accurate data collection. The prone position used in the experiment is just one example, and in this example, the original axes of the sensor are located at the initial position aligned with the directions of gravity (minus *z*-axis of the sensor) and geomagnetism (*x*-axis of the sensor). Besides, we put the finger joint at the edge of the table to avoid the movement of the proximal phalanx so as to reduce the errors of its position measurement.

Once the sequence of rotation matrices _2_^1^**R**_*i*_ is obtained through the above tests, the joint axis of the PIP joint can be computed. Similarly, by placing one additional sensor on the distal phalanx, the joint axis of the DIP joint can be determined.

In the experiment, the flexion-extension movements were continuously repeated 3 times during one test process. The results obtained from the above tests are processed and illustrated in Figure 5.  Figure 5(a) shows the results for the PIP joint, and the blue line clusters are the direction vectors of PIP joint axis obtained from each rotation matrix _2_^1^**R**_*i*_ during the rotation process, which indicates that the joint axis direction varies slightly at each. The red line indicates the average direction vector of the rotation axis of the PIP joint. From the figure, it can be found that presented in the coordinate frame {*O*_*p*_}, for the PIP joint in the index finger, the average direction vector of the joint axis is ${\bar{\omega }}_{\text{PIP}}={\left[\begin{array}{ccc} 0.998 & 0.024 & 0.061 \end{array}\right]}^{T}$ with around ±3.5° variation, of which the variation of the joint axis is the maximum angle between the average joint axis vector (red line) and each instantaneous joint axis vector (blue line). The maximum angle was identified by using the embedded MATLAB command. Similarly, presented in the coordinate frame {*o*_*m*_}, for the DIP joint, the direction vector of the joint axis is ${\bar{\omega }}_{\text{DIP}}={\left[\begin{array}{ccc} 0.955 & 0.231 & 0.184 \end{array}\right]}^{T}$ with around ±5° variation. Accordingly, a 14° orientation difference can be found between the average rotation axes of PIP and DIP joints. The result is consistent with the description of the cadaveric tests presented in Ref. [4, 6].

Further, using the screw displacement transformation derived in Section 2.2, based on the rotation axes of the PIP and DIP joints in an index finger identified above, motion of the distal endpoint with respect to the PIP joint can be formulated and characterised. Let us define the natural anatomical position as the reference (zero) position, give the screw axes of the PIP and DIP joints as **ω**_PIP_ = **ω**_2_ = (0.998, 0.024, 0.061) and **ω**_DIP_ = **ω**_3_ = (0.955, 0.231, 0.184) as identified from the above in vivo tests, and specify the lengths of the middle and distal phalanges as *l*_2_ = 23.16 mm and *l*_3_ = 15.83 mm, respectively. Forward kinematics of the distal and middle phalanges relative to the PIP joint can be formulated as

(30) $$\begin{array}{c} T_{O_{p}O_{d}}=e^{\left[S_{2}\right]\theta_{2}}e^{\left[S_{3}\right]\theta_{3}}M_{O_{d}}, \end{array}$$

where in coordinate frame {*O*_*p*_}, there are **S**_2_ = (**ω**_2_, **r**_2_ × **ω**_2_) with **r**_2_ = (0, −*l*_2_, 0) and **S**_3_ = (**ω**_3_, **r**_3_ × **ω**_3_) with **r**_3_ = (0, −(*l*_2_ + *l*_3_), 0) and **M**_*O*_*d*__, and the position vector of point *o*_*d*_ in the zero configuration expressed in the reference frame {*O*_*p*_} as

(31) $$\begin{array}{c} M_{O_{d}}=\left[\begin{array}{cccc} 1 & 0 & 0 & 0\\ 0 & 1 & 0 & -l_{2}-l_{3}\\ 0 & 0 & 1 & 0\\ 0 & 0 & 0 & 1 \end{array}\right]. \end{array}$$

Substituting the parameters into Eqs. (24) and (30) and using the experimental joint angle range of the PIP and DIP joints from [15] as *θ*_2_ ∈ [0, 101°] and *θ*_3_ ∈ [0, 73°], workspace of the fingertip (i.e., point *o*_*d*_) can be calculated and plotted as shown in Figure 6. One can see that the workspace is distributed in a three-dimensional space rather than on a plane. This workspace is generated due to the offset of the axes of rotation of the PIP and DIP joints from their anatomical planes, which leads to the conjoint rotation, and thus the three-dimensional motion of the fingertip.

## 4. Discussions

From the above derivation and investigation, we found that the rotation axes of the PIP and DIP joints are offset from the anatomical planes, such an arrangement leads to conjoint rotations [1] that generate three-dimensional motion for dexterous grasping and manipulation of hand with fewer joints. The axes of rotation of the PIP and DIP joints are not fixed but vary throughout the range of motion of the joints. This agrees with the statements in [19, 20]. As pointed out in [20], the finger joints are synovial joints which move with both rotation and sliding, and, hence, the axes of rotation are the evolute of the serial of locations of the instantaneous axes of rotation. In clinical practice and in ordinary clinical situations [1], simplification to an average axis of rotation, like formulated in Eq. (29), is assumed to occur throughout the entire range of motion of a joint. This average direction of axis is located by an anatomic landmark that pierces the convex member of the two bones forming the joint. The results obtained by the proposed method in this paper also agree with the experimental results in [21], which indicates that the PIP and DIP joint axes are not fixed, the joints are approximately parallel to the flexion-extension creases [1, 2], and are approximately perpendicular to the bone segments in full extension, but progressively are oblique during flexion. The MR image measurement in [4] showed changes of up to 14° in the directions of the PIP and DIP joint axes during motion. In [22], based on the 3D scanned data, the changes of axes of rotation of finger joints during motion were characterised as surface of screws based on screw theory, and the results are similar to those illustrated in Figure 5 in this paper. In addition, we found that the proposed method was more efficient than the “axis finder” [2]. If we want to identify the rotation axes of the MCP joint in both flexion-extension and abduction-adduction planes, the “axis finder” system needs to be reconstructed to find the rotation axis in different planes. But using the proposed gyroscope sensor, we can keep the same position of the sensors to identify all the rotation axes in one joint.

Further, the experimental results obtained in this paper have some errors because of the noise in the sensor's signals and the deformation of the finger tissue and skin during the movement. In addition, the rotation axis direction in the finger joint can be quite different between individuals, and, thus, for clinical and medical applications, the test needs to be carried out individually. The above experimental setup, testing process, and data processing method hence provide an efficient, convenient, and intuitive approach for identifying rotation joint axis in human fingers. This approach is efficient for not only the PIP and DIP joints in the fingers and IP joint in the thumb, but also the MCP and CMC joints. In order to identify the joint axis vectors of the DIP, PIP, and MCP joints in the fingers at the same time, the additional sensors need to be placed on the distal, middle, and proximal phalanges and the metacarpal bone. Otherwise, two sensors are enough for one joint axis identification even there are more than one degree of freedom. These will be investigated in our future research.

Therefore, in this paper, a low-cost, efficient, and intuitive in vivo approach is proposed for detecting axes of rotation of the PIP and DIP joints of the index finger. Using the proposed method, rotation axes of the one degree of freedom joints in the hand can be conveniently identified. The method can be extended to the identification of axes of rotation of PIP and DIP joints of the other fingers and IP joint of the thumb, and it can be also potentially extended for determining axes of rotation of the other synovial joints, such as knee joint and elbow joint, in the human body.

## 5. Conclusion

Kinematics and axes of rotation of human joints are important in constructing prosthetic joints and planning reconstructive surgery, and, hence, various methods including goniometry, mechanical finder, MR and CT images, and surface markers have been used to identify the axes of rotation of joints, especially finger joints. In this paper, a low-cost, intuitive, and portable in vivo method based on gyroscope sensors was for the first time proposed for detecting axes of joints of the PIP and DIP joints in an index finger. The proposed experimental method was integrated with screw displacement representation of rigid body motion, and the matrix exponential-based derivation of general spatial displacement was described in a detailed manner, providing background for wider applications in the field of biomechanics. The experimental results demonstrated the efficiency and effectiveness of the proposed method, and the results are comparable and agree with the previous published works [4, 6].

## Figures and Tables

**Figure 1:** Rotation of rigid body 1 about the axis **ω** by an angle *θ*.

**Figure 2:** Geometry of general spatial displacement of a rigid body.

**Figure 3:** (a) Coordinate frames attached to each phalanx of a finger; (b) rotation of the middle phalanx about the PIP joint with respect to the proximal phalanx.

**Figure 4:** Gyroscope sensor in in vivo test of joint axis of PIP joint in an index finger.

**Figure 5:** The rotation axes in PIP and DIP joints in an index finger.

**Figure 6:** Workspace of the fingertip with respect to frame {*O*_*p*_} based on the identified rotation axes of the PIP and DIP joints in an index finger.

## Data Availability

No data are associated with this paper.
